# Anomaly Detection in Videos Using Two-Stream Autoencoder with Post Hoc Interpretability

**DOI:** 10.1155/2021/7367870

**Published:** 2021-07-26

**Authors:** Jiangfan Feng, Yukun Liang, Lin Li

**Affiliations:** ^1^Chongqing University of Posts and Telecommunications, School of Computer Science and Technology, Chongqing, China; ^2^Chongqing Geomatics and Remote Sensing Center, Chongqing, China

## Abstract

The growing interest in deep learning approaches to video surveillance raises concerns about the accuracy and efficiency of neural networks. However, fast and reliable detection of abnormal events is still a challenging work. Here, we introduce a two-stream approach that offers an autoencoder-based structure for fast and efficient detection to facilitate anomaly detection from surveillance video without labeled abnormal events. Furthermore, we present post hoc interpretability of feature map visualization to show the process of feature learning, revealing uncertain and ambiguous decision boundaries in the video sequence. Experimental results on Avenue, UCSD Ped2, and Subway datasets show that our method can detect abnormal events well and explain the internal logic of the model at the object level.

## 1. Introduction

The video's abnormal event detection is to find events different from usual, such as people fighting or urgent events like fire. It is an essential task in the computer vision field, from both academia and industry. As video cameras continue to expand, exploiting video data is currently severely limited by the amount of human effort, so that the automatic detection of rare or unusual incidents and activities in a surveillance video is urgently needed [1]. Although abnormal event detection has inspired plenty of works based on computer vision techniques [2–4], it is still quite challenging to design a general detection framework because of the definition uncertainty and limitations of the data-generating mechanism.

Deep learning technologies have been widely used to detect abnormal events, including unsupervised methods [5, 6] and weakly supervised methods [7]. Recently, another developing approach for video processing in the deep learning framework is two-stream networks, which have been successfully applied to video-based action recognition [1, 4], often with state-of-the-art results. Despite the excellent performance, none of these methods considers the black-box problem brought by deep learning models. Regarding practical use, to ensure the proposed method can produce reliable results, a model's interpretability is required.

Advances in computer vision have led to an interest in automated computational methods for video surveillance. The anomaly detection task [5–12] mainly trains a regular model with only normal samples and then marks the samples in the test dataset different from the normal samples. Recently, more and more approaches have employed deep learning [5–7, 12–20] to learn the features of the video frame. Those methods train the model to get better detection results. For instance, Ravanbakhsh et al. [17] proposed combining CNN high-level semantic information and low-level Optical-Flow as a new method of measuring anomalies.

Besides, Feichtenhofer et al. [3] proposed to use SlowFast Networks for video recognition. SlowFast networks can be described as a single stream architecture that operates at two different frame rates. In contrast, we use the two-stream autoencoder network to learn features and generate the reconstructed video sequence to detect anomalies. Tudor Ionescu et al. [10] first proposed to use unmasking to deal with learned characteristics. Different from our method, it is to use a binary classifier to determine anomalies. Fan et al. [11] proposed the Gaussian Mixture Variational Autoencoder, which used the Gaussian Mixture Model (GMM) to fit the distribution of the feature space through the variational method. Sabokrou et al. [13] proposed a cubic-patch-based way containing 3D deep autoencoders and 3D convolutional neural networks for an advanced feature-learning approach. Luo et al. [18] proposed to combine Convolutional Long Short-Term Memory (Conv-LSTM) with Autoencoder to learn the appearance and action information of the video. The model will output the reconstructed sequence input at the current time and last time. Chong and Tay [20] proposed an effective method for video anomaly detection, which is suitable for the spatiotemporal structure of video anomaly detection, including crowded scenes.

Herein, we propose an unsupervised learning scheme to detect abnormal events using a novel two-stream network by utilizing late fusion, with its inherent logic through post hoc interpretability: (1) We propose an abnormal event detection algorithm in surveillance video that offers a potential improvement on two key elements, that is, the interpretability and the performance of detection, which is of great significance in video surveillance. (2) The proposed two-stream architecture learns the appearance characteristics of the video through a spatial model, and the temporal model is a temporal autoencoder to learn the regular pattern in the video. The advantage is the suitability of modeling the spatial characteristics using relatively few training samples. (3) We visualize the feature map of the convolution layers and outputs the features learned by the convolution layers at the object level through a heatmap, enabling abnormal object detection. Furthermore, it helps users identify essential features of surveillance tasks, demonstrate the importance of features, and reproduce the decisions made by the black-box model.

## 2. Related Work

Applying the method of interpretable deep learning to anomaly detection is an emerging research direction, and it is still in the development stage. The extension includes two significant aspects.

### 2.1. Semantics of the CNN

Although CNNs have achieved significant momentum in computer vision tasks, the end-to-end learning strategy brings about infrequent interpretability [21]. On the other hand, it can help ensure impartiality in decision-making and provides a truthful causality in model inference [22]. The visualization of filters in CNNs is the most direct way to explore the visual patterns hidden in neural units. Firstly, most visualizations are gradient-based methods [23–27]. These methods mainly calculated the gradient scores of convolutional neural network units and used them to evaluate the image's appearance to maximize its unit fraction. Similar approaches, up-convolutional networks [28], were a typical way of visualizing the representations of CNNs. Besides, Zhou et al. [29] provided a method to precisely calculate the neural activation image receptive field. However, these methods are postinterpretation of online learning, which did not adjust the model or affect the final decision.

Apart from neural network visualization methods, machine learning models can also explain neural networks. Some approaches focused on learning networks with disentangled representations to represent the semantic hierarchy hidden inside CNNs [30, 31]. Zhang et al. [32] proposed a quantitative interpretation of convolutional networks' prediction logic through decision trees. This method can learn explicit representations of object parts in the high convolutional layers of CNNs while mining potential decision modes in fully connected layers. Besides, Zhang et al. [33] proposed modifying CNNs by adding a loss to each filter of a high convolutional layer to receive the deentanglement representation. Wu et al. [34] proposed an interpretable localized convolutional neural network for object detection. These interpretation methods are different from network visualization. In particular, a previous study [35, 36] showed the potential of interpretable deep learning techniques for predicting properties of simulated low-dimensional magnetic systems.

### 2.2. Abnormal Event Detection

Previous studies in abnormal event detection have suggested that the detection model can be trained from the reconstruction task. Hasan et al. [7] introduced a full autoencoder with manually annotated data, and anomaly detection was based on reconstruction loss. Luo et al. [16] used time-coherent sparse coding to encode two adjacent frames with similar reconstruction coefficients. However, the abnormal events observed in these models were primarily dependent on reconstruction error. As a result, it might fit abnormal events unexceptionally. Thus, the prediction model compared the predicted frame with the actual video frames for anomaly detection. GANs are usually used to enhance the predictive ability [37–40]. Moreover, constraints in motion and gradient are also proven effective. Liu et al. [41] proposed a framework based on future frame prediction to detect anomalies. However, the prediction method can be sensitive to noise and perturbation, especially in scenes with illumination changes, leading to inferior robustness in anomaly detection. Thus, Qiang et al. [42] proposed an anomaly detection model based on the latent feature space, combining the above two methods. In addition to detecting abnormal events from learning-based techniques, Yu et al. [43] proposed a neuromorphic vision sensor, a natural motion detector for abnormal objects. Recently, several authors have presented abnormal video detection by the two-stream convolutional network. Simonyan and Zisserman [44] proposed a two-stream network to recognize the actions of video objects. Kingma and Welling [22] proposed a new fusion method based on the two-stream structure to identify the action information in the video. They found that spatial and temporal networks can be fused in the convolutional layer but not in the softmax layer. Subsequently, Yan et al. [1] proposed a two-stream abnormal detection method, and the model is composed of an appearance stream and action stream.

However, most of the video abnormal event detection algorithms cannot achieve online monitoring. The first difficulty is that the model has many layers, the structure is more complex, and detecting anomalies is too time-consuming. Therefore, we want to learn spatial-temporal features through the two-stream network and learn features through some relatively lightweight architectures, but the detection performance can also be excellent. Besides, none of these deep methods considers the “black-box” characteristics, and it demonstrates the urgent need to apply the internal logic of anomaly detection at the semantic level. Therefore, we want to show the most critical features of surveillance tasks and reproduce the decisions made by the black-box model.

## 3. Proposed Method

The general workflow for our method (Figure 1) includes two streams (spatial stream and temporal stream), which learn features during the encoding stage, and then generate reconstructed sequences of the raw video sequence through decoding. The method can be considered as unsupervised learning scheme in which an autoencoder is trained on the normal data through reconstruction. If an abnormal event occurs, the corresponding reconstruction error score is higher than the normal data since the model has not met the irregular pattern during training. Besides, we visualized the spatial model's convolutional layer features to identify ways that could help further understand and display the process of model learning at the object level to help people comprehend and trust the detection results of our model.

### 3.1. Autoencoder-Based Reconstruction

The input to the two-stream network is regular video frames. We trained the model, and the reconstruction error was calculated between the initial and reconstructed frames. Reconstruction error is used to calculate the regularity score that can be further evaluated for the detection performance of the system. Our approach generates reconstruction errors from both the spatial and temporal streams in the testing stage and then fuses them appropriately.

Our approach contains three main steps.

#### 3.1.1. Preprocessing

The various video clips were used to build and test our model, which differed in size, shooting time, and definition. We decomposed the anomaly detection datasets into a sequence of video frames and unified the video frame size to 224 × 224 pixels. To ensure that the input video frames are all on the same scale, we computed the training image's pixel average. Then, we subtracted each frame from the average global image for normalization. We also converted the image to grayscale to reduce the dimensionality. Because of the large number of learnable parameters and limited given training datasets, we used data augmentation [7] to enlarge the training data set in the temporal dimension. The enlargement is done by generating the new cuboids with various skipping strides to construct *T*-sized original video frames (for example, In stride-1 cuboids, all *T* frames are consecutive, whereas, in stride-2 and stride-3, cuboids skip one and two video frames, respectively).

#### 3.1.2. Feature Learning

We used a spatial stream to learn the appearance and used a temporal stream to learn the temporal coherency on adjacent video frames. The temporal model consists of three parts, the convolution layers, the deconvolution layers, and the convolution long short-term memory (Conv-LSTM) layers. The convolutional layer is used to learn each frame's spatial or behavioural characteristics. The deconvolutional layer is used to restore the original input size, and the Conv-LSTM layer outperforms the temporal rules of the video. Our spatial model is similar to the temporal model, but the spatial model lacks a Conv-LSTM layer, and its input is in the form of a single frame instead of consecutive frames.

*(1) Spatial Model*.  Figure 2 shows the detailed configuration of the proposed spatial model. It only consists of three convolutional layers, followed by two deconvolutional layers to improve efficiency. Since anomaly detection focuses more on low-level contours, edge features, the spatial model only uses three convolutional layers for feature extraction. On the other hand, the role of the deconvolutional layer is to generate reconstructed video frames and densify the sparse inputs by operations with multiple filters. Hence, the spatial size of the output feature maps of a deconvolutional layer is larger than the spatial size of its corresponding inputs. Therefore, we extract the person's appearance feature in the video through the three-layer convolution layer and restore the initial input dimensions through the connected two deconvolution layers. The parameters are designed to balance the strength of the convolutional and deconvolutional layers. Therefore, we optimize them alternatively with the layer-parameter set through the training process. During the training stage, the learnable parameters were updated toward the direction minimizing the loss function. We used MSE loss based on the Relu function. By calculating the partial derivatives of the loss function, we could update the parameters in an SGD scheme.

The feature-learning process is the essential stage of model training. In the encoding stage, the model learns the spatial features of the monitored object in the video frame and the critical background information in the monitored scene. Also, the spatial model architecture and input are relatively simple. The feature map visualization algorithm is to transparentize the “black box” of the spatial model, understand the model's learning process, and trust the final detection results.

*(2) Temporal Model*. The temporal model may have similarly formulated but different layers based on LSTM requirements. To better learn the temporal coherency on adjacent frames, we added three layers of Conv-LSTM between the convolution layers and deconvolution layers (Figure 3). The dimensions of the three layers are the same, and the main difference is the number of convolution kernels.

The input to the temporal model is the video volume. Considering the effect of frame length on model training and memory consumption speed, we chose four consecutive frames with various skipping strides in this paper. The frame number is a trade-off parameter in learning. This length of training on the subway dataset is just what our machine can meet, and the speed of training and testing was relatively good. Shi et al. [45] proposed the Conv-LSTM model first, and Patraucean et al. [46] utilized the model to predict the next video frame. To extract both temporal and spatial features of the Conv-LSTM model, we inputted the image as *X*, and a convolution filter replaces the set of weights for each connection, which can get the timing relationship and extract the spatial features like the convolutional layer.

#### 3.1.3. Reconstruction Error

After we got the reconstructed sequence of the video frame, we calculated its reconstruction error between the initial video frame and the reconstructed frame to model standard data's probability distribution. In our proposal, reconstruction is a stochastic process that considers the distance between the reconstruction and the initial video frame and the variability of the distribution itself. To qualitatively analyze whether our model can detect anomalies well, we used the regularity score graph to indicate the ability of our model to detect anomalies. The regularity score corresponds to the level of normality of each frame in the video.

In practice, we first counted the reconstruction error of the video frame before getting the regularity score sr(*t*). Then, we calculated the reconstruction error of the pixel intensity value *I* at the location (*x*, *y*) in frame *t* as follows:

(1) $$\begin{array}{c} p\left(x,y,t\right)={\left\|I\left(x,y,t\right)-f\left(I\left(x,y,t\right)\right)\right\|}_{2}, \end{array}$$

where *f* represents our two-stream model. We calculate the Euclidean distance between the initial pixel of the *t*-th frame and the pixel of the reconstructed frame as the reconstruction error of the pixel. For each frame, we compute the reconstruction error probability by summing up all the pixel-based probabilities.

(2) $$\begin{array}{c} R\left(t\right)=\sum_{\left(x,y\right)}p\left(x,y,t\right). \end{array}$$

After calculating the reconstruction error of the spatial model *R*_*S*_(*t*) and temporal model *R*_*T*_(*t*), respectively. We calculated the reconstruction error of the fusion model *R*_*F*_(*t*). Due to the different dimensions of the two models. The fused reconstruction error *R*_*F*_(*t*) can be obtained using the following equation:

(3) $$\begin{array}{c} R_{F}\left(t\right)=R_{S}\left(t\right)*R_{T}\left(t\right). \end{array}$$

After we define the reconstruction error probability of a frame as *R*_*F*_(*t*), the abnormality score can be defined as follows:

(4) $$\begin{array}{c} S_{a}\left(t\right)=\frac{R_{F}\left(t\right)-\min_{t}R_{F}\left(t\right)}{\max_{t}R_{F}\left(t\right)-\min_{t}R_{F}\left(t\right)}. \end{array}$$

The abnormality score *S*_*a*_(*t*) corresponds to the level of abnormality of each frame in the video, which plays a role in indicating the confidence of detection results. On the other hand, the regularity score *S*_*a*_(*t*) corresponds to the level of normality can be defined as follows:

(5) $$\begin{array}{c} {\text{s}}_{r}\left(t\right)=1-s_{a}\left(t\right). \end{array}$$

Assume that the regularity score of the current frame is relatively low. In this case, the possibility of abnormality in the video frame is high. On the other hand, if there is no abnormality in the video frame, the regularity score of the frame should also be relatively high.

### 3.2. Feature Map Visualization Algorithm

This algorithm is based on the visualization of the feature map in CNNs, transforming the image's interior features into a visible and understandable image pattern, which helps us clearly understand the features learned by the model. The feature learning of convolutional neural networks is an incomprehensible process for humans to confirm whether it has learned features that have a natural effect on prediction, for example, in detecting abnormal events, whether it judges or predicts an abnormality based on understanding the abnormal behaviour characteristics of the monitored object. After extracting each convolutional layer's features, the model generated a certain number of feature maps. We can use the visual feature map to explain the features learned by the model in each convolutional layer, helping us understand and trust the final result. Inspired by Grad-CAM [26], we combined the feature map of the convolutional layer with the input image to generate the heatmap and display the features learned by the model's convolutional layer in the form of objects in the heatmap. Compared with other studies, the main difference in our work performs the reconstructed video sequence that does not need to get the gradient of the convolutional layers. Therefore, we directly superimposed the feature map into the abnormal frame in the form of a heatmap without changing its gradient. The method proposed in this paper can realize visual feature maps in any convolutional layer in spatial and temporal models and has particular applicability in deep learning models in other fields.

Assuming that the current convolutional layer of the model has *n* feature maps, the convolutional layer here can be any layer, denoted as *A*^1^, *A*^2^,…, *A*^*n*^, the size of the feature map is *r∗c*, *S*=*r∗c*.The pixel values of the *k*-th row and the *j*-th column of the *i*-th feature map are *A*_*kj*_^*i*^. The activation mapping *LAM* for this layer is as follows:

(6) LAM=ReLU ∑i=1nwi∗Ai,Ai=1S∑k=1r∑j=1cAkji,LAM=ReLU 1S∑i=1n∑k=1r∑j=1cwi∗Akji.

Among them, *w*_*i*_ corresponding to the weight of each neuron, the value is 1 in this paper. Because the spatial model is based on the Autoencoder, it learns the characteristics of many monitored objects in the video frame. Unlike the object classification task, the video anomaly detection task needs to learn the features of all objects. Therefore, each feature map may contain multiple object parts, adding each feature map in a one-to-one ratio. Using the ReLU function is that only the part with the feature value greater than 0 is needed, that is, the part that the model focuses on.

### 3.3. Abnormal Detection

This method combines the feature map visualization algorithm with the two-stream network to solve the low reliability of the deep learning model in video anomaly detection. When abnormal events were detected, the internal logic of the model was explained through a heat map. Thus, the method was divided into two parts: (1) anomaly detection based on a two-stream network; (2) visualization based on the heat map. The two parts can operate independently or put together.

The anomaly detection process can also be divided into two parts (Figure 4): (1) merge the spatial flow network and the temporal flow network to detect anomalies; (2) use a separate subnetwork to learn features to detect anomalies. Both parts need to preprocess the video, decompose the video clip into video frames, learn the features, reconstruct the video frame, and calculate the frame's regularity score. Temporal and spatial networks are autoencoders, and they can generate reconstructed frames through reconstruction methods and calculate regularity scores. Because the inputs of the two networks are different, the spatial model was input in a single video frame, which reduced the memory consumption of model training. The temporal model needs to model the correlation between adjacent video frames, so the Conv-LSTM layer was used and input in four video frames. The advantage of the model design was that relatively few training samples were used to model spatial features, and learned spatial and temporal features were separated through two submodels. Then, the two models can be fused to achieve better anomaly detection results. In addition, the model design is relatively simple, which improves the speed of learning and finding anomalies. Through model fusion, the detection performance can be guaranteed within a reasonable range.

## 4. Experiment and Results

### 4.1. Datasets

We conducted experiments on four public benchmark datasets: Avenue [47], UCSD, Ped2 [48], and Subway Exit and Entrance datasets [49]. The Avenue dataset has 16 training video clips and 21 test video clips. The duration of each clip varies from less than one minute to two minutes. The UCSD Ped2 dataset is where pedestrians move parallel to the camera plane, containing 16 training and 12 test videos. The Subway Entrance video is 1 hour and 36 min long and consists of 66 abnormal events, while the Subway Exit dataset includes 19 abnormal events, and the duration is 43 minutes. Since the subway video clips are too long and the amount of data is too large, we only used the first 5 minutes of the Subway Exit video for training and the first 15 minutes of the Subway Entrance video. Then, the test dataset is divided into 4 and 6 test videos. Each test video is a continuous segment, and the approximate duration is 10 minutes and 13 minutes, respectively. (The former is the Subway Exit dataset; the latter is the Subway Entrance dataset.) Table 1 shows the details of the datasets.

### 4.2. Model Configuration

Here, we provide a detailed configuration of our method in Table 2. Moreover, all experiments running on a PC equipped with a GeForce RTX2080 GPU, 64G RAM, and running the Windows 10 operating system.

### 4.3. Experiment on Anomaly Detection

#### 4.3.1. Quantitative Analysis: Frame-Level AUC

To better compare with other methods, all the experiments are carried out on the same PC with Intel CPU I7 8700K, NVIDIA GTX 2080, and 64G RAM. If a frame contains at least one abnormal event, it is considered as a correct detection. This detection is compared to the frame-level ground-truth label. The area under the curve (AUC) and the equal error rate (EER) are the evaluation's two metrics. Furthermore, some contemporary documents [9, 10] believe that the EER evaluation criteria are a severe sample imbalance between normal and abnormal events. Using EER as an indicator will be misleading in practical applications. We agree with this view and use AUC for evaluation, assuming that the local minimum within 50 frames belongs to the same abnormal event.

*(1) Effectiveness Analysis*.  Table 3 presents the AUC of our method and a series of state-of-the-art methods [7, 10–12, 14, 18, 20] on the Avenue, the UCSD Ped2, and the Subway Entrance and Exit datasets. As expected, our model performs the best performance on the avenue and subway entrance and exit datasets. In addition, although the version in Avenue and Ped datasets appears to be slightly lower than that in the other complicated architectures, it is still significantly higher than that of lightweight models and that single-level models. These results indicate that a multilevel model [14] or 3D indicator [12] can perform better in crowd-scene, such as the UCSD Ped2 dataset. However, the time cost of these methods was also higher. Besides, comparing our spatial model and temporal model and the fusion model, temporal and spatial model have their advantages and disadvantages. Still, the fusion model performs better than the former two on all data sets.

*(2) Time-Cost Analysis*. Besides the effectiveness analysis, we also compare the computation time cost of the proposed approach. Since the proposed methods are based on the reconstruction techniques with deep learning, the model during the test is compared with other reconstruction-based deep methods.  Table 4 shows the average computation time of different deep ways. Only four video frames in the temporal stream and a single video frame in the spatial stream generate the reconstruction error in our process. Thus, less time is needed for reconstruction error computation. The result shows the proposed approach is comparable with other methods.

#### 4.3.2. Qualitative Analysis: Visualizing Frame Regularity

The regularity score graphs obtained by the spatial and temporal models are similar, so only the spatial model's regularity scores are shown. Figures 5–8 illustrate the regularity score of each frame on the Avenue, UCSD Ped2, Subway Entrance, and Exit video, respectively. When an anomaly is detected, the regularity score of the anomaly frame is significantly decreased. Further, our model can also detect unlabelled abnormal events.

Although our training process only used the usual scenes in the data set, our method can detect abnormal events that do not appear in the ordinary scene (Figure 5). For example, people enter the subway station from the subway station's exit for some prominent abnormal events and then enter and take the subway from here. As can be seen from the figures, the detection results match well with the ground-truth frames. The lower regularity scores correspond to abnormal events, while high regularity scores correspond to regular video frames. In the regularity score graph, the blue line is the regularity score of the video frame, and the red part is the abnormal event occurrence area marked by the ground truth. In Figures 5–7, according to the ground-truth anomaly labels, we can easily find abnormal events by setting the threshold to 0.5, excluding any false-positive detection. However, in some scenarios, false-positive detection will occur when the threshold is set to 0.5.

To better analyze the performance of our method, we also plot the anomaly score from Avenue, Ped, and Subway datasets. Figures 9–12 provide the detected events and the corresponding anomaly scores on the related data sets, with the anomaly score curve of the spatial, temporal, and two-stream fusion. The peak color regions indicate the frame-level ground-truth label of abnormal events. As can be seen from the figures, the detection results match well with the ground-truth frames.

### 4.4. Post Hoc Interpretability with Feature Visualization

Besides the quantitative and qualitative analysis, we use a heatmap to visualize the features of abnormal behaviour, such as skateboarding on the sidewalk, or entering the subway without playing, etc. Since the first three layers of the model's learned features are similar, this paper only shows the visualized heatmap of the first convolutional layer.

Figures 13–16 provide different visualization of the same data and show the features of the first convolutional layer on the Avenue dataset, UCSD Ped2 dataset, Subway Entrance, and Exit scenes, respectively. The frames are containing abnormal events and ordinary events. We achieve comparable results with the other two leading methods, and comparison experiments show that our method can detect anomalous objects well.  Figure 13 shows our model learns a specific behaviour characteristic of people, such as losing the packet or walking around. As the running person is too fast, detecting abnormal behaviour characteristics is not so obvious.  Figure 14 shows that our model is more interested in pedestrians walking and riding bicycles or carts. As shown in Figures 15 and 16, our model is interested in the people and characteristics of the track or train. These features can help our model identify the subway entrance and exit scene and the two videos' anomalies. In contrast, Grad-CAM [26] only visualizes some abnormal object regions, and Grad-CAM [27] visualizes many abnormal object regions.

Figures 13–16 show that our model can learn visual appearances and motion in the scene, helping to understand images and infer abnormal events. For example, Figure 13 shows an example illustrating the appearance and contour of vehicles with a darker color. Similarly, Figure 16 shows a person jumping over the fence and entering the subway exit. Thus, the model learns that the visual impressions and behaviours of individuals, combined with the scene. Therefore, it can be concluded that an abnormal event has occurred here. Therefore, our feature map visualization experiment can also verify the accuracy and authenticity of the abnormal detection results. Besides, the visualization method can explain the learning process of the model, but the visualization result will not affect the learning process and the final detection. Therefore, the interpretation method of this article can be considered as post hoc interpretability.

Conceptually, abnormal events are emerging from uncommon objects. Thus, while visualization of a trained model provides insight into its operation, it can also assist with selecting anomalous objects in abnormal video frames. The critical question is if the model identifies the object's location in the image with unnatural object detection approaches.

### 4.5. Discussion

Our results suggest that the proposed method enables fast and reliable detection of abnormal events, with label-free identification of abnormal events. In the quantitative experiment introduced in 4.3.1, we used four video frames in the temporal stream and a single video frame in the spatial stream to generate the reconstruction error, while number frames preferring ten were most frequently used by other methods. Using only the spatial or temporal stream cannot cause the best result. However, with the information from the two-stream fused, the model has improved efficiency compared with a single stream, while the accuracy is also competitive. It should also be noted that our current model is lightweight and does not consider the complete appearance and motion of the video scenario. Therefore, the training process in our method does not reconstruct all the changes in the properties of appearance and motion, and it may be weak compared with other techniques in a particular dataset—for example, GMFC-VAE in Ped2.

Compared with other anomaly detection methods [5, 6, 16–20], we use a heat map to visualize the internal logic of the video frames, which is more interested in the darker part. Therefore, we can better understand the network's learning process and the basis for making abnormal behaviour judgments. We also compare the visualization of feature maps of different convolutional layers. Due to the relatively small number of layers, we find the features learned by the first and second convolutional layers are almost the same. They are relatively low-level edge and contour information rather than high-level abstract details. Our method exhibited interpretability and much better location stability than other anomaly detection methods.

In summary, these results highlight the effectiveness and high efficiency of the proposed method in abnormal event detection. However, although it can show interpretability in abnormal event detection, it is challenging to present interpretable loss terms in end-to-end training.

## 5. Conclusions and Future Work

We have presented a prevailing method to detect abnormal events from videos to intensify detection ability and feature interpretability with a two-stream framework. Our approach fuses the visual appearances, behavioural characteristics, and motion of the video object and can determine abnormal events from many regular activities. To critically assess the robustness of detecting in capturing abnormal events, we performed several challenging data sets that allow our algorithm to operate robustly for long periods in various scenes, including crowded ones. Experiments have shown that our method is accurate and robust to noise. Furthermore, the visualization of feature maps semanticizes the internal logic.

Meanwhile, applying explainable deep learning methods to anomaly detection will be a future research direction. It has excellent benefits for handling abnormal events and even preventing abnormal events from happening in advance, which has great significance in public security.

## Figures and Tables

**Figure 1:** The pipeline of our method. First, we need to decompose the video of datasets into continuous frames. Then we use the convolutional two-stream network to learn the feature of image frames. Finally, the video frame's regularity score is calculated to decide this frame is normal or abnormal. From the initial image to the heatmap, we can see that the model is more interested in areas where abnormal events occur, such as the patrol car that appears here.

**Figure 2:** Spatial model architecture. The rightmost number indicates the output size of each layer.

**Figure 3:** Temporal model architecture. The final output is the reconstructed frame sequence.

**Figure 4:** Anomaly detection flowchart. The first step is to process the video, learn the features through the two-stream network, and calculate the reconstruction error to detect anomalies.

**Figure 5:** Regularity score of video #5, #7, and #15 from the Avenue video.

**Figure 6:** Regularity score of videos #2, #4, and #7 from the UCSD Ped2 video.

**Figure 7:** Regularity scores of frames 15000–30000 and 45000–57500 from the Subway Exit dataset.

**Figure 8:** Regularity score of frames 20000–40000 and 80000–100000 from the Subway Entrance dataset.

**Figure 9:** Anomaly score of videos #5, #7, and #15 from the Avenue video.

**Figure 10:** Anomaly score of videos #2, #4, and #7 from the UCSD Ped2 video.

**Figure 11:** Anomaly scores of frames 15000–30000 and 45000–57500 from the Subway Exit dataset.

**Figure 12:** Anomaly score of frames 20000–40000 and 80000–100000 from the Subway Entrance dataset.

**Figure 13:** Feature visualization results on our method, Grad-CAM, and Score-CAM on Avenue dataset. Top-3 rows are abnormal video frames, and the last row is a normal video frame. (a) Initial video frame. (b) Our method. (c) Grad-CAM. (d) Score-CAM.

**Figure 14:** Feature visualization results on our method, Grad-CAM, and Score-CAM on UCSD Ped2 dataset. Top-3 rows are abnormal video frames, and the last row is a normal video frame. (a) Initial video frame. (b) Our method. (c) Grad-CAM. (d) Score-CAM.

**Figure 15:** Feature visualization results on our method, Grad-CAM, and Score-CAM on Subway Entrance dataset. Top-3 rows are abnormal video frames, and the last row is a normal video frame. (a) Initial video frame. (b) Our method. (c) Grad-CAM. (d) Score-CAM.

**Figure 16:** Feature visualization results on our method, Grad-CAM, and Score-CAM on Subway Exit dataset. Top-3 rows are abnormal video frames, and the last row is a normal frame. (a) Initial video frame. (b) Our method. (c) Grad-CAM. (d) Score-CAM.

**Table 1:** Details of the datasets.

Dataset	Frames	Training frames	Testing frames
Subway	125475	22500	102975
UCSD Ped	18560	9350	9210
CUHK Avenue	30652	15328	15324

**Table 2:** The parameter settings of our method.

Parameter	Value
Height	160
Width	240
Batch size	16
Lr	0.01
Epoch	200
Optimizer	SGD
Stride	4
Loss	MSE

**Table 3:** Comparison of area under ROC curve (frame-level AUC) of different methods.

Method	Avenue	Ped2	Subway Entrance	Subway Exit
ST-AE [20]	76.5	81.7	81.8	86.4
Unmasking [10]	80.6	82.2	70.6	85.7
GMFC-VAE [11]	78.6	84.9	83.7	87.4
RBM [12]	78.7	86.4	—	—
DAEs + cGAN [14]	73.6	86.1	84.1	87.3
ConvAe [7]	74.3	79.7	84.9	83.9
Conv-LSTM-AE [18]	76.4	82.9	83.3	86.4
Spatial model	78.1	83.8	84.7	90.2
Temporal model	77.8	84.0	85.0	85.4
Spatial + temporal	80.3	84.5	87.3	90.8

Higher AUC is better.

**Table 4:** Comparison of the average computation time (per epoch) on four data sets.

Method	Avenue (m)	Ped2 (m)	Subway Entrance (m)	Subway Exit (m)
ST-AE [20]	180	30	640	360
ConvAe [7]	244	40	320	120
Conv-LSTM-AE [18]	312	73	766	452
GMFC-VAE [11]	220	65	712	432
DAEs + cGAN [14]	430	194	904	642
Spatial model	19	3	24	8
Temporal model	95	15	120	50
Spatial + temporal	142	24	182	70

## Data Availability

The data used to support the findings of this study are available from the corresponding author upon request.
